# Analysis of Political Subjective Initiative and the Construction Path of Advanced Education from the Network Community Environmental Perspective

This article has been retracted.

**DOI:** 10.1155/2022/7034414

**Published:** 2022-08-03

**Authors:** Wen Zhang

**Affiliations:** College of Marxism, Xi'an Jiaotong University, Shaanxi 710049, China

## Abstract

According to the data of the Research Report on online communities, the current online communities and the interaction between members rely on major platforms. Among them, WeChat has a relatively high degree of use, which can reach 61.1%, followed by self-built apps, which are used by 52.8% and 50.0%, respectively, providing a good communication space for community members. Users' viscosity to the network is increasing, which makes users more dependent on the network. This is undoubtedly a squeeze for politics and advanced education. Therefore, based on the upgrading of education positions, ensuring the effectiveness of education puts forward higher requirements for the construction of education paths in the network community environment. Through the analysis of the topic map of social network public opinion users, models with different dimensions are built, so as to provide an effective theoretical basis for education and ensure the healthy development of online community environmental education.

## 1. Introduction

Technological progress has promoted social development, but the penetration of the network in various fields of society has also changed people's thinking and way of life. Based on this background, the network community, which has both technical and social attributes, is a micro mapping of the new social form [1]. For the current people, the iterative updating of network community types and how to ensure the concentration of users' thoughts, actively play the role of political and advanced education, and explore the effective path of education from the perspective of the community are of great significance to the current society and the development of the network community. Based on the relationship between individuals and groups, this paper deeply analyzes social relations, discusses the development of social networking, and constructs a guiding mechanism suitable for the collaborative management of users' online communities, which has a practical impact on modern ideological education [2].

The progress of technology is an important driving force to promote the changes of the times and the evolution of social forms. The progress of network technology is not only widely influencing and promoting the innovation and development in various fields of economy and society but also profoundly changing people's living conditions and development methods [3]. The development of network technology has further promoted the interaction between people, and the social structure and form have changed accordingly. As shown in Figure 1, after the increase in the number of Internet users, the Internet is not a technological reform but a revolution in society and human relations. With the progress of scientific and technological means, online communities are becoming more and more developed, and students are more accustomed to contacting, communicating, and receiving educational information through online communities. The education of subjective initiative is also completed through the network to a greater extent. This kind of political education completed by the online community environment is more convenient and promotes low carbon development to a greater extent and reduces the environmental burden.

Facing the ideological and political education and advanced education in the new era, we need to face the connotation characteristics of the network community, so as to investigate the relationship between people and society and accurately grasp the characteristics of the network in the new era. Only in this way can a more effective network-based community be formed to provide users with correct education. In this regard, how can the connotation of online community be understood? How can the group usage on the user network be explored? In the face of the new era of network development, how to accurately grasp the new characteristics and changes of the behavior and thought of educational objects and explore new educational paths is the primary problem we are facing [4]. For a modern society, education in the network era is more conducive to accurately grasp the elements of network development and make effective responses according to its development and change rules. Secondly, it is more helpful to promote the innovation of ideological education practice. It can optimize the content construction of the educatees' online community according to the understanding of the educational objects, so as to promote and optimize the construction of the online community and provide more effective guidance for education.

## 2. The Spreading Mode and Evolution Mechanism of Knowledge in Network Community

### 2.1. Definition of Knowledge in the Network Community Environment

Knowledge is an essential factor in knowledge transmission. Previous researchers defined knowledge as the organization and refinement of the information obtained to solve practical problems, the improvement of personal ability, and the establishment of personal interaction network. According to the definition of scholars and the background of knowledge development, knowledge refers to the processing and integration of information, data, and other resources, which are applied to the solution of practical problems or the accumulation of personal capital. Compared with the characteristics of common substances that will be continuously lost and depreciated in the case of repeated use, knowledge is a constant value-added in the process of use [5]. Especially in the online community environment, knowledge is spread more widely and shared more frequently, and knowledge shows greater value in the process of superposition and interaction of community members.

### 2.2. Knowledge Dissemination Mode under the Network Community Environment

The existence of communication mode connects various elements together. For the current knowledge communication, there are three types: hierarchical communication, tower communication, and network communication [6].

#### 2.2.1. Hierarchical Communication

As shown in Figure 2, it can be seen that the hierarchical communication mode is divided into different levels. In the process of communication, both the disseminator and the receiver complete the corresponding behavior under the condition of anonymity, but, as a social person, the individual will be affected by both personal and environmental factors in the whole process of communication activities, which will bias his knowledge communication behavior.

#### 2.2.2. The Tower Communication Mode of Knowledge Constructed from the Perspective of the Communicator

As shown in Figure 3, it can be found that knowledge dissemination in the online community environment is no longer limited by time and space, and the boundary between the disseminator and the receiver is eliminated. Therefore, the disseminator and the receiver can be unified as participants in knowledge dissemination, and the positioning of the receiver can be weakened. Building a knowledge dissemination model based on knowledge contribution can also highlight the equality of the knowledge dissemination process. Through the use of more open media, knowledge contributors' contributions to knowledge continue to stack, which also illustrates the expansion of knowledge dissemination in depth in the online community environment [7].

#### 2.2.3. Network Communication Mode of Knowledge Constructed from the Perspective of the Recipient

In the process of communication, different network environments lead to different user knowledge networks. Users will build a knowledge network according to their own needs. Based on the good interaction between individuals in the overall network structure, they can effectively contribute knowledge to others.  Figure 4 shows the network knowledge model. The knowledge dissemination mode in the network community environment has the characteristics of multiple layers and nesting. In this system, there are three types of structural holes, which are, respectively, attached to the three-tier network. The knowledge energy exchange between structural holes ensures the mutual mapping between the three-tier networks and forms a personal knowledge system network through the process of knowledge transmission [8].

### 2.3. Analysis of Knowledge Evolution Stages in Online Communities

The online community has low threshold access and strong liquidity. It is an open system. The relationship between members is loose and fragile and will change constantly. In order to maintain the stable and balanced development of the whole system, it needs to inject energy into it continuously. The dissemination of knowledge in the network community will not be a fixed model, and the evolution of knowledge under the framework of this model is also a dynamic process.

First, we need to ask questions based on knowledge formation and select and integrate according to their own knowledge needs to help the whole evolution process be activated. Second, the network community provides an energy storage platform for the evolution of knowledge, so that the value of knowledge will not be exhausted, and knowledge can form a knowledge base through continuous self-accumulation. When the critical point of knowledge spillover occurs, the breadth of knowledge will be deepened and the content branch will be fuller. Thus, a huge knowledge base is formed, and users can collect almost all relevant content in the system by means of retrieval, inquiry, link, or sharing [9]. At this point, the diffusion of knowledge has a great influence on the network community platform and is concerned and discussed by more users, thus gradually entering the next stage. This stage belongs to the peak of knowledge transmission, which can attract extensive attention and discussion, so that the positive and negative views begin to cluster and evolve into the peak. Finally, knowledge in the online community is formed after precipitation and feedback. In this process, the evolution of knowledge did not end but entered a new evolution process through the continuous interaction between users and knowledge, between users, and between users and platforms, so as to ensure the sustainable existence of the vitality of the network community. As shown in Figure 5, the evolution of knowledge in online communities seems complex, but in fact there are certain laws. Only by finding the existing laws can we strengthen the interaction between the platform and users and enter the new knowledge evolution cycle [10].

### 2.4. Mechanism of Knowledge Dissemination in Online Communities

The emergence of network community has subverted the previous knowledge communication mode, making the subject of knowledge communication shift. The participation and release, sharing and collaboration, and integrated feedback of knowledge dissemination are integrated into the same platform by the online community, which provides a strong platform support for knowledge dissemination and establishes a personal centered community-based knowledge dissemination mechanism. Through this mechanism, the accessible area of knowledge dissemination is wider, the coverage is wider, and the content of knowledge dissemination is deeper, which improves the efficiency of knowledge dissemination and shortens the knowledge radius among members. As shown in Figure 6, it can be seen that knowledge dissemination is in a circular mechanism, and the structure is relatively stable [11]. Among them, the participation release mechanism mainly refers to the use of personal knowledge to transfer to the organization into organizational knowledge. The sharing and cooperation mechanism is the mutual transformation of knowledge between users and between users and platforms, so as to realize knowledge interaction, cooperation, coconstruction, and symbiosis. The integrated feedback mechanism is to transfer the information provided by users to the community platform for correction and verification or to rectify in the internal organization through collective wisdom, so as to invest in a new round of knowledge participation and release closed-loop process mechanism [12].

## 3. Social Network Public Opinion User Theme Map System Model

### 3.1. Composition of Social Network Public Opinion User Theme Community Map

#### 3.1.1. Information Ecological Elements of Social Network Public Opinion User Theme Map

The social network public opinion user topic map system model is closely related to the information ecology theory, and the knowledge map can visually analyze the elements of the information ecology. This section focuses on the analysis of the four elements of information ecology of the topic map of social network public opinion users, that is, environmental elements, subject elements, object elements, and technical elements. Based on the four mentioned elements, the mechanism of information ecology element model is described [13]. The environmental factors of the social network public opinion user theme map are shown in Figure 7.

#### 3.1.2. Main Elements of Social Network Public Opinion User Theme Map

The main elements of the topic map of public opinion users in social networks correspond to the informants in the information ecosystem. This refers to public opinion users who use the corresponding information technology to express their views, emotions, propositions, and attitudes by publishing public opinion information in a certain social network public opinion space. In the main elements of the social network public opinion user theme map, the information person classification is represented by ellipse, and the information role classification is usually represented by rectangle.  Figure 8 shows the processing flow of the user unit.

#### 3.1.3. Information Ecological Element Model of Social Network Public Opinion User Theme Map

In the topic map of social network public opinion users, the information environment, informant, information, and information technology together constitute the information ecosystem of the topic map of social network public opinion users. Environmental elements, subject elements, object elements, and technical elements are the four information ecological elements of the theme map of social network public opinion users [14]. The information ecology element model of social network public opinion user theme map is constructed by information technology, as shown in Figure 9.

#### 3.1.4. Construction of Social Network Public Opinion User Theme Map

The entity in the social network public opinion user topic map refers to the basic unit carrying information in the social network public opinion information environment. For its understanding, as shown in Figure 10, according to the attributes and concepts represented by different nodes, different edges in the graph represent the relationship between different semantics. Each node can have one or more attributes. The identification of user information needs the support of relevant algorithms to solve the redundancy caused by information overload. An effective entity recognition method is the basis for constructing the topic map of social network public opinion users. From the development process of entity recognition technology, the current mainstream methods include rule-based entity recognition method and machine-learning-based entity recognition method, which can also be used in combination [15]. The accuracy of the rule method is high, but it is difficult to achieve because of cost factors, and rule onfa does not have the ability of horizontal migration. Compared with the rule-based implementation, the machine learning method has better robustness and flexibility and does not need too much manual intervention or additional prior knowledge. However, machine learning methods rely on large-scale training data, which cannot effectively solve the problem of sparse data, and some methods have poor convergence [16].

### 3.2. Composition of Social Network Public Opinion User Theme Map

Based on the relevant theories of information ecology and knowledge map, this paper mainly makes an in-depth study from three aspects: The first is how social network public opinion user topic map contributes to community discovery, user identity, and emotional evolution. The second is that, at the same time, information makes the informant form a certain influence in the information environment. The third is that information technology, as the main technical support, ensures the accuracy, timeliness, and security of information circulation [17].

#### 3.2.1. Social Network Public Opinion User Community Map

In a specific public opinion space, due to the differences of public opinion users' own information resources and information culture, they will gather into different network communities, thus forming different community environments. Only by combining the agent model can we further understand the user community map, discover the relationship between communities, and effectively identify the user characteristics and other elements [18].

#### 3.2.2. Social Network Public Opinion User Identity Map

Based on the identity and communication characteristics of informants, this paper uses information technology to analyze the life cycle of public opinion and analyzes the process of informants' participation during this period. The user identity is classified and the evolution process is analyzed. Classification algorithm is used for user identification and establishing visual atlas. Different from the static portrait description based on registration information, the identification of social network public opinion user identity map is based on the analysis of users' public opinion information under different topics, which can intuitively present the public opinion relationship between different users.

#### 3.2.3. Social Network Public Opinion Ecology and Evaluation

In the research process, according to the analysis, a comprehensive evaluation index system is constructed from the four dimensions of community information environment, users, technology, and emotion to explore the symbiotic law between various elements. The relationship among environment, subject, object, and technology in social network public opinion is effectively interpreted. The ecological nature of social network public opinion mainly studies the systematic law of the interaction of ecological constituent elements and observes whether there is a positive interaction between different constituent elements and whether it promotes the benign operation of the whole ecosystem. The ecological evaluation based on the user theme map of social network public opinion has changed the traditional analysis method of social network public opinion and information ecology. By analyzing its ecological evolution logic, it is clear that the long-term and stable development of social network public opinion ecology depends on the interaction of its participating elements under certain time and space conditions, as shown in Figure 11 [19].

Horizontally, the public opinion space corresponding to the information environment can deeply mine the network community in the space. Information corresponds to public opinion information, and the emotional tendency of public opinion information can be analyzed through the user's emotional map. Vertically, the information environment includes the informants in the environment, and each informant is the direct producer of information, which is a research process from macro to micro level. Public opinion space contains different public opinion users, and public opinion users are the main providers of public opinion information in the public opinion space, which is a research process from the whole to the specific [20].

## 4. Social Network Public Opinion User Community Map Construction and Community Discovery

Based on the theory of information ecological environment, combined with the LDA theme model of JS divergence, the social network public opinion user community map is constructed, and the community relationship is found. Based on social topics, the user's theme preference is analyzed. User community map is used to identify user characteristics.

### 4.1. Raising Problems

With the increasing popularity of the network, users' information interaction in the network community becomes more frequent. The network is made to become an amplifier of social public opinion. On the other hand, traditional analysis methods mostly use calculation indicators for identification, resulting in the inundation of small-scale communities. By constructing the social network public opinion user community map, we can tap the potential themes of the community, divide the network community, and determine the community theme preference. It is the key to ensuring the coordinated development of public opinion and plays a certain guiding and reference role for public opinion supervision [21].

### 4.2. Social Network Public Opinion User Community Discovery Model

#### 4.2.1. LDA Subject Model

Latent Dirichlet allocation (LDA) is a generative model, which is essentially a multilevel Bayesian probability graph model. This probability graph model contains three granularity structures: document, topic, and word. The core idea is that each document corresponds to a word that obeys the Dirichlet distribution $\bar{\theta }$, and each topic corresponds to a word that obeys the Dirichlet distribution $\bar{\phi }$, where the document topic distribution *α* parameter and the topic word distribution *β* parameter obey the Dirichlet distribution and $\bar{\alpha }\text{ and }\bar{\beta }$. In the field of machine learning, the topic model plays an important role. The optimal number of topics is determined through the confusion evaluation index. The formula is as follows:

(1) $$\begin{array}{c} \text{perplexity}n\;Dn=\exp\frac{\sum_{d=1}^{M}\log\;nW_{d}n}{\sum_{d=1}^{M}N_{d}}n\;\ln\;, \end{array}$$

where *D* represents the set of all words in the document, *M* represents the number of documents, *W*_*d*_ represents the words in document *D*, *N*_*d*_ represents the number of words in each document, and *P* (*W*_*d*_) represents the probability of words in the document. The degree of confusion generally decreases with the increase of the number of potential topics. The smaller the degree of confusion, the stronger the ability of the topic model. Therefore, this chapter selects values with relatively low confusion and relatively small number of topics as the optimal model parameters for LDA topic model training.

#### 4.2.2. Similarity Measurement

After obtaining the optimal number of topics through the confusion degree, the document topic distribution can be obtained through the LDA topic model. After obtaining the document topic distribution matrix, this chapter uses JS (full name: Jensen Shannon divergence) to calculate the topic similarity between users and uses it as the edge weight in the construction of community map. JS divergence measures the similarity of two probability distributions and is a variant of KL (full name: Kullback-Leibler divergence). Since KL divergence is not symmetrical, it is not conducive to the construction of downstream community map. JS divergence effectively solves the problem of asymmetric KL divergence, and its value is between 0 and 1 [22]. The calculation formula is as follows:

(2) $$\begin{array}{c} JSnP\|Qn=\frac{1}{2}KLnPnxn\|\frac{Pnxn+Qnxn}{2}+\frac{1}{2}KLnQnxn\|\frac{Pnxn+Qnxn}{2}nn2n,\\ KLnP\|Qn=\sum Pnxn\;\log\frac{pnxn}{Qnxn}n3n. \end{array}$$

In the above formula, *P*(*x*) and *Q(x)* represent the probability distribution of users with different public opinions, that is, the document topic distribution obtained by LDA topic model. If there are *m* pieces of user information, the topic distribution is *m∗n*, and a square matrix of *m∗m* is obtained to obtain the division of public opinion users. Through this similarity measure, we can find the nearest neighbor user set and determine the network community in the information environment [23].

### 4.3. Construction of Social Network Public Opinion User Community Map Model

Social network public opinion user community map is built based on LDA topic model. The user community map model built in this chapter is shown in Figure 12. After the JS divergence is calculated, the user community map is constructed with the public opinion users of the common theme as the node and the JS divergence as the edge weight information, and the network community is divided and the corresponding characteristics of the community are analyzed.

### 4.4. Data Collection and Analysis

In this chapter, Python is used to collect the keywords published by public opinion users according to the content shown in Figure 13. The advanced search function is used to crawl all pages in a request and store them. XPath parsing is used to obtain user related information. Jump to the next level request according to the time when the text is published [24].

After data processing by access and excel, the invalid fields and contents in the data are normalized to make the text topic incline towards a more original direction. To determine the optimal topic, we need to train the text classification after processing. The integer within the range of 2 to 30 is proposed as the number of topics, and the logarithm confusion value of different models is obtained by calling the log_perplexity method under the LDA topic model class, as shown in Figure 14. The horizontal axis in Figure 14 shows the number of potential topics in the LDA topic model, and the vertical axis shows the confusion degree of the LDA topic model. The broken line in the figure shows that, as the number of topics increases, the overall degree of confusion shows a fluctuating upward trend. The local minimum of confusion degree appears in the model selection with the number of topics being 7. According to the Occam's razor criteria mentioned above, and in order to ensure that the model covers differentiated topics as much as possible, this chapter intends to select 7 as the topic parameter value of LDA topic model.

After the optimal topic is selected, the text data needs to be processed. The distribution of each topic is shown in Table 1.

As can be seen from Table 1, the probability values of keyword occupation of each topic are relatively large, which conforms to the characteristics of the text topic. Even if users have different comment habits, they can also divide topics by model. It can be found that most public opinion users' forwarded comment texts have obvious topic division, and the topic tendency of public opinion users can be effectively mined through LDA topic modeling.

### 4.5. Social Network Public Opinion User Identification Model

The sampling process of LDA subject model should follow the core idea of Dirichlet model. That is, assuming that *M* pieces of microblog public opinion information are collected, totaling *n* words, and the number of topics of microblog information is *k*, the sampling process of LDA topic model is as follows: select a parameter according to the collected topic distribution, and generate *N* keywords according to the steps. The keywords are assigned according to the parameters and distributed to the corresponding topics. Thus, according to the distribution of randomly generated topics, the generated words are obtained.

In order to better control public opinion, most microblog platforms have introduced the identity discrimination dimension, so that the algorithm can realize the identity screening mechanism. The user identity needs to be authenticated. The user identity features are

(3) $$\begin{array}{c} \text{Identity}=\text{verify}+\log\;ne^{\text{follower}-\text{following}}+e^{\text{num}}n. \end{array}$$

“Verify” indicates whether the user has passed the authentication mechanism of the microblog platform. “Follower,” “following,” and “num” are the number of fans, followers, and tweets, respectively. *Z*-score normalization is required before the formula is brought in. The formula is *Z*=(*x* − *μ*/*σ*), where *x* is the characteristic value to be specified, *μ* is the mean value, and *σ* is the standard deviation.

The construction of communication features is defined as follows: propogatinon=log  *ne*^follower^+*e*^repost^+*e*^comment^*n*+like, where “follower,” “repost,” “comment,” and “like” correspond to the number of followers, forwarding, comments, and likes, respectively, and the value is obtained after *Z*-score normalization. The promotion value is proportional to its propagation ability. The larger the value, the stronger the propagation ability.

### 4.6. Naive Bayesian Classifier

As a generative model, naive Bayesian classifier estimates the posterior probability from the prior probability based on the assumption of attribute conditional independence and Bayesian formula. Information *D* is abstracted into a word bag model, which is a document composed of *n* words *w*, defined as *D*={*w*_1_*nw*_2_*n* … *nw*_*n*_}, and the user category belongs to *C*={*c*_1_*nc*_2_*n* … *nc*_*n*_}. Based on the assumption of attribute condition independence, the user identity classification calculation should be $c_{NB}=\arg\underset{c_{i}\in C}{\max Pnc_{j}n\prod_{i=1}^{n}Pnw_{i}|c_{j}nc_{i}}$. The prior probability of *Pnc*_*j*_*n* user category can calculate the known information. Based on the given category conditions, the conditional probability is calculated such as the formula *Pnc*_*j*_*n*=(Doc*nc*_*j*_*n*/∑_*c*_*j*∈*C*__Doc*nc*_*j*_*n*). The posterior probability is calculated as follows:

(4) $$\begin{array}{c} Pnw_{i}nc_{j}n=\frac{\text{Weight}nw_{i}nc_{j}n}{\sum_{i=1}^{n}\text{Weight}nw_{i}nc_{j}n}. \end{array}$$

It should be noted here that when category *C*_*j*_ in the text is missing, the calculation result is 0. In view of the limited amount of information and the difficulty in forming a sample space, the formula is improved to eliminate the negative impact of the 0 factor, and the formula is improved to

(5) $$\begin{array}{c} Pnw_{i}nc_{j}n=\frac{\text{Weight}nw_{i}nc_{j}n+\delta }{\sum_{i=1}^{n}\text{Weight}nw_{i}nc_{j}n+\delta \left|V\right|},\\ V=\sum c_{j}\in C\sum_{i=1}^{n}\text{Weight}nw_{j}nc_{j}nn\delta =\frac{1}{\left|V\right|}. \end{array}$$

### 4.7. Overview of Public Opinion Events and Cycle Division

In order to better divide the public opinion life cycle, it is necessary to analyze the node event probability of information. As shown in Table 2, according to the time stage, the event cycle can be divided into three cycles: outbreak, spread, and recession. According to the characteristics of the event, the topic heat increases. After the user's participation, the topic gradually enters the recession period. It can be seen from the classification results of social network public opinion users' identities that, according to the statistics of user identity types, the participation process of various types of public opinion users can be mastered. Media public opinion users have a high degree of participation in each public opinion life cycle and have the right to speak about most public opinion topics. Public opinion users in the aviation industry have significant participation at most key time points but quit the discussion during the recession. The participation of relevant enterprise nodes in Manyan is high, which once exceeded that of the media. The participation of ordinary people in the whole life cycle of public opinion has been relatively stable.

## 5. Conclusion and Prospect

Under the background of network community, the era of community has been formed in the process of political initiative and Progressiveness Education and in the network technology of weeding out the old and bringing forth the new. Looking back at the rise, formation, and development of online communities, there is no doubt about the crucial importance of technology driven, but it is not the only decisive factor. This research has always been guided by the awareness of the above problems, placed the research under the macro background of information technology reform, the rise of the network society, and human survival and development, followed the research philosophy of “technology human (individual group)—society,” and made every effort to conduct a multiangle and multidimensional investigation on the intrinsic connotation of the network community and the deep-seated causes, internal and external drives, and value significance of the formation and development. It brings some enlightenment for the ideological and political education to explore the appropriate response path and highlight the vitality in the online community.

This paper attempts to explore and put forward some practical paths for ideological and political education to integrate into the network community and play an educational and guiding role in the network community, starting from the objective dimensions of enhancing the embeddedness, communication, and guarantee of the network community of college students' ideological and political education. However, due to the sustainability of technological innovation and social change, in order to promote the effective “implementation” of relevant measures in practice and give full play to the vitality of political education in online communities, it is still necessary to continuously track and refine research in combination with practice. This also provides the impetus for the author to continue to carry out in-depth and expanded research around this topic and field in the future.

## Figures and Tables

**Figure 1:** Size of Internet users and Internet penetration in China.

**Figure 2:** Knowledge level communication mode.

**Figure 3:** Tower mode of knowledge transmission.

**Figure 4:** Knowledge network model.

**Figure 5:** Analysis of knowledge evolution stages in online communities.

**Figure 6:** Knowledge dissemination mechanism in online communities.

**Figure 7:** Environmental elements of social network public opinion user theme map.

**Figure 8:** User unit's processing flow.

**Figure 9:** Ecological element model of social network public opinion user theme map.

**Figure 10:** Knowledge map < entity relationship > concept map.

**Figure 11:** Ecological evolution logic of social network public opinion user theme map.

**Figure 12:** Social network public opinion user community map model based on the LDA topic model.

**Figure 13:** User publishing content and platform.

**Figure 14:** Line chart of permeability topic.

**Table 1:** Distribution of clustering subject high frequency words.

Subject 0	Pilot	Crash	Release	Ethiopia	Responsibility
Probability	0.0.31	0.022	0.021	0.042	0.032
Topic 1	Grounded	Fault	Publish	China	Global
Probability	0.038	0.032	0.016	0.013	0.012
Topic 2	Photo	Passport	Staff	Accident	Information
Probability	0.028	0.026	0.015	0.016	0.016
Topic 3	Publish	Video	Status	Rummage	Maneuver
Probability	0.027	0.024	0.021	0.020	0.019
Topic 4	Press conference	China Eastern Airlines	Air China	Relics	Girl
Probability	0.044	0.036	0.036	0.030	0.020
Topic 5	Boeing	System	Defect	Aircraft	Aircraft
Probability	0.062	0.039	0.039	0.038	0.037
Topic 6	Family members	Victim	Prosecution	Dead	Remains
Probability	0.019	0.016	0.017	0.015	0.015

**Table 2:** Event probability of key event nodes.

Time	Key events
2019/03/10	Cause the accident
2019/03/12	News release from multiple countries
2019/03/14	Arrival of relatives of the victims of the accident
2019/03/29	Investigation report released
2019/04/12	Official response

## Data Availability

The labeled dataset used to support the findings of this study is available from the corresponding author upon request.
